# Prediction and Screening Model for Products Based on Fusion Regression and XGBoost Classification

**DOI:** 10.1155/2022/4987639

**Published:** 2022-07-31

**Authors:** Jiaju Wu, Linggang Kong, Ming Yi, Qiuxian Chen, Zheng Cheng, Hongfu Zuo, Yonghui Yang

**Affiliations:** ^1^College of Civil Aviation, Nanjing University of Aeronautics and Astronautics, Nanjing 210016, China; ^**2**^ Institute of Computer Application, China Academy of Engineering Physics, Mianyang 621900, China

## Abstract

Performance prediction based on candidates and screening based on predicted performance value are the core of product development. For example, the performance prediction and screening of equipment components and parts are an important guarantee for the reliability of equipment products. The prediction and screening of drug bioactivity value and performance are the keys to pharmaceutical product development. The main reasons for the failure of pharmaceutical discovery are the low bioactivity of the candidate compounds and the deficiencies in their efficacy and safety, which are related to the absorption, distribution, metabolism, excretion, and toxicity (ADMET) of the compounds. Therefore, it is very necessary to quickly and effectively perform systematic bioactivity value prediction and ADMET property evaluation for candidate compounds in the early stage of drug discovery. In this paper, a data-driven pharmaceutical products screening prediction model is proposed to screen drug candidates with higher bioactivity value and better ADMET properties. First, a quantitative prediction method for bioactivity value is proposed using the fusion regression of LGBM and neural network based on backpropagation (BP-NN). Then, the ADMET properties prediction method is proposed using XGBoost. According to the predicted bioactivity value and ADMET properties, the BVAP method is defined to screen the drug candidates. And the screening model is validated on the dataset of antagonized Er*α* active compounds, in which the mean square error (MSE) of fusion regression is 1.1496, the XGBoost prediction accuracy of ADMET properties are 94.0% for Caco-2, 95.7% for CYP3A4, 89.4% for HERG, 88.6% for hob, and 96.2% for Mn. Compared with the commonly used methods for ADMET properties such as SVM, RF, KNN, LDA, and NB, the XGBoost in this paper has the highest prediction accuracy and AUC value, which has better guiding significance and can help screen pharmaceutical product candidates with good bioactivity, pharmacokinetic properties, and safety.

## 1. Introduction

The inherent reliability of the equipment depends on the reliable design of the product. Therefore, before the electronic components are installed on the whole machine or equipment, it is necessary to try to eliminate the problematic components as much as possible. Therefore, it is necessary to screen the components based on the performance prediction value for improving the reliability of the equipment system. Similarly, drug screening is to inspect and test substances that may become drug products and predict their properties based on inspection and test values, to find drug values and clinical uses, and to provide data and data support for the research and development of new drugs. Drug discovery is a high-cost, high-risk process. According to Pharmaceutical Research and Manufacturers of America (PhRMA) statistics, it takes an average of 10 to 15 years and costs $2.6 billion for each drug to go from early discovery to Food and Drug Administration (FDA) approval. Despite this, PhRMA statistics find that the US biopharmaceutical industry's investment in new drug discovery is still gradually rising, from $15.2 billion in 1995 to about $90 billion in 2016 [1]. It can be seen that in the entire drug discovery process, the cost and time consumption of the clinical stage is huge, but the throughput is small [2]. In other words, the economic loss brought by stopping the development of the drug in the clinical stage is huge. Therefore, how to improve the success rate of drug discovery and identifying drug candidates that may fail at an early stage is a problem that pharmaceutical companies have been trying to overcome [3–5].

The main reasons for the failure of contemporary drug research and development are the low bioactivity of the candidate compounds and the deficiencies in their efficacy and safety, which are related to the absorption, distribution, metabolism, excretion, and toxicity (ADMET) of the compounds [6, 7]. At present, in vitro or in vivo experiments are mainly used to test these properties of compounds. However, due to species differences, these methods are costly, time-consuming, and often difficult to extrapolate from in vitro to in vivo or from animals to humans. On the other hand, the current performance optimization of ADMET properties mainly relies on expert experience, which partly comes from the knowledge of chemical biology and partly from the summary of previous experiments [8], but it is ultimately limited. With the production of more and more experimental data and the development of computer technology, we pay more and more attention to finding laws and building models to predict and optimize compounds in a data-driven way. The use of computational models is not only low cost, but to some extent, it may be more accurate than experiments and smarter than humans [9, 10]. At the same time, related technologies such as machine learning are increasingly being used to predict the screening of compounds with specific pharmacodynamics and ADMET properties, which has promoted drug discovery and evaluation [11].

Establishing a compound activity prediction model is usually used to screen potential active compounds. The common method is to collect a series of compounds that act on the target and their bioactivity data for a target related to the disease and then use a series of molecular structure descriptors as independent variables to determine the dependent variable and bioactivity value, constructing the quantitative structure-activity relationship (QSAR) model [12], and then use the model to predict new compound molecules with better bioactivity or to guide the structure optimization of existing active compounds [13]. In the actual QSAR model, the value is experimentally measured and usually has a positive correlation with bioactivity, that is, the greater the value, the higher the bioactivity. In addition, for a compound to become a drug candidate, in addition to having good bioactivity, it also needs to have good pharmacokinetic properties and safety in the human body, collectively known as ADMET [14]. Among them, ADME mainly refers to the pharmacokinetic properties of the compound, which describes the law of the concentration of the compound in the organism over time, and *T* mainly refers to the toxic and side effects that the compound may produce in the human body. No matter how good a compound's bioactivity is, if its ADMET properties are poor, for example, it is difficult to be absorbed by the human body, or the metabolism rate in the body is too fast, or it has some toxicity; then it is still difficult to be a candidate drug, so ADMET properties also need to be predicted and optimized. Usually, to facilitate modeling and prediction, it is regarded as the binary classification method; 1 means good properties, while 0 means poor. However, the prediction accuracy is low, causing the screening for drug candidates still be inefficient and high-cost [15].

Therefore, we propose the prediction and screening model for drug candidates based on fusion regression and extreme gradient boosting (XGBoost) and verify it on the data set that can antagonize estrogen receptors *α* (Er*α*) compounds. We use the fusion regression, which is the light gradient boosting machine (LGBM) for further feature extraction and BP-NN to predict bioactivity value and XGBoost binary classification to predict the ADMET properties. And the verification results show that the XGBoost works better than other methods. Based on the predicted bioactivity value and ADMET properties, we can use the bioactivity value and ADMET properties (BVAP) method to quantitatively screen drug candidates, which can improve the success rate of drug candidates screening and guide the drug screening process.

The rest of this paper is organized as follows: Section 2 introduces the related work on the prediction of bioactivity value and ADMET properties.  Section 3 introduces the prediction and screening model.  Section 4 introduces the verification and experiment.  Section 5 introduces the conclusion, some limitations, and the future expansion of the paper. Finally, some patents are declared, and relevant references are provided.

## 2. Related Work

Lei et al. [16] used six machine learning methods to establish the prediction model, including relevance vector machine (RVM), support vector machine (SVM), regularized random forest (RRF), extreme gradient boosting, naive Bayes (NB), and linear discriminant analysis (LDA). Erić et al. [17] explored artificial neural network (ANN) and SVM ensemble-based models, as well as knowledge-based approaches to descriptor selection. Jiang et al. [18] used seven machine learning methods including a deep learning method, two ensemble learning methods, and four classical machine learning methods to build classification models. Nayarisseri et al. [19] provided an overview based on some applications of machine learning based tools for drug identification, QSAR modeling, and ADMET analysis. Zhang et al. [20] summarized the history of machine learning and provided insight into recently developed deep learning approaches in rational drug discovery. Cheirdaris [21] provided an overview of the applications of artificial neural networks (ANNs). Yang et al. [22] developed PySmash to generate different types of representative substructures for safety evaluation. Hessler and Baringhaus et al. [23] put forward ANNs such as recurrent neural networks (RNNs) for drug discovery. Raju et al. [24] integrated in silico approaches to identify selective inhibitors. Lei et al. [25] developed a series of QSAR models for predicting urinary tract toxicity. Dobchev et al. [26] gave an overview of the strategies and current progress in using machine learning methods for drug design. Hsiao et al. [27] have applied machine learning methods for classification as well as regression analysis to a publicly available intravital data set to assess the intrinsic metabolic clearance in humans. These results suggest the usefulness of machine learning techniques to derive robust and predictive models in the area of intravital ADMET modeling. Their suggestions provided ideas for our research. Kovalishyn and Poda [28] reported the batch pruning algorithm for variable selection. They combined the ANN ensemble learning and self-organized map of Kohonen for clustering of descriptors. Gola et al. [29] considered advances in statistical modeling techniques for predictive ADMET models in drug discovery. Sun et al. [30] performed a QSAR and classification study based on a total of 134 base analogs related to their ED50 values. Li et al. [31] trained five machine learning classifiers, that is, K-nearest neighbor (KNN), SVM, random forest (RF), XGBoost, and DNN on each feature set of histone deacetylase 3 to facilitate prospective screening for inhibitors. Zhang et al. [32] used the genetic algorithm to select important molecular descriptors and used the NB for the in silico prediction model.

According to the current research of related work, data-driven methods such as machine learning are increasingly applied to predict bioactivity value and ADMET properties. It can be divided into two aspects.

On the one hand, when screening potential active compounds, the main methods are ANN and other basic machine learning algorithms, such as GA, MLP, and RFSA. In this paper, we first use LGBM to mine further features inside the data and use BP-NN, that is, ANN based on backpropagation, to predict bioactivity value more accurately.

On the other hand, when predicting the ADMET properties, the main methods are SVM, RF, KNN, NB, LDA, and their transformations. In this paper, we use XGBoost to predict ADMET properties. The advantages and disadvantages of the above methods are shown in Table 1.

However, few papers are researching the bioactivity value and the ADMET properties simultaneously and combining them into one model. The screening model we proposed could predict both of them to help screen pharmaceutical product candidates with good bioactivity, pharmacokinetic properties, and safety.

## 3. Model and Methods

The pharmaceutical products screening model is divided into four parts, and the flowchart of this model is shown in Figure 1.

It can be seen from Figure 1 that first, we do data preprocessing according to the preprocessing rules, and then it can be the input for parts 2 and 3. In part 2, we use the fusion regression to predict the bioactivity value. For part 2.1, we use LGBM for further feature extraction to get the molecular descriptors related to the bioactivity value. For part 2.2, we the molecular descriptors to predict the bioactivity value. In part 3, we use XGBoost to predict ADMET properties. In part 4, we propose a new BVAP method to screen drug candidates. The model can screen drug candidates with better bioactivity value and ADMET properties, thereby effectively serving the screening and preparation for drug candidates.

### 3.1. Data Preprocessing

The molecular descriptor is a quantitative description symbol for drug molecules' structure and physical-chemical properties. Usually, molecular descriptors are robust, or there is a high linear correlation between molecular descriptors, so an appropriate subset of molecular descriptors should be extracted from them to make the model have better predictive ability. Therefore, to remove low-information variables or redundant variables, the following steps are used:

1. If the relative variance of a molecular descriptor is less than *σ*, delete the molecular descriptor
2. If the correlation coefficient of a pair of molecular descriptors is greater than *C*, delete any one of the molecular descriptors

Here, *σ* and *C* are constants that need to be defined. Generally, the larger the relative variance, the higher the information variables; the larger the correlation coefficient, the higher the redundancy between the data. Therefore, we need to delete the molecular descriptor with low relative variance and high correlation coefficient.

### 3.2. Quantitative Prediction with Fusion Regression

In this part, the fusion regression assembles the LGBM and BP-NN to make the quantitative prediction. The LGBM is used to extract the further features related to the bioactivity value and also reduce the dimension of the BP-NN input layer, thereby reducing the complexity of its training; the BP-NN is to use the extracted features to predict the bioactivity value.

#### 3.2.1. LGBM for Feature Extraction

LGBM is a gradient boosting framework based on the classification and regression tree. The negative gradient of the loss function is used as the approximate residual value of the current subtree to fit the new subtree. Its advantage is that while retaining large gradient samples, it randomly retains some small gradient samples and at the same time amplifies the information gain brought by small gradient samples.

In terms of feature extraction, LGBM optimizes the support for category features. It can directly input category features without additional expansion. LGBM uses the basic idea of the gradient boosting decent tree to measure the importance of the feature by using the total number of times the feature is used to split in all decision trees [33]. Then the features are sorted in descending order by importance, and the search is started from the complete set of sample features. According to the accuracy of the result, it is judged whether to remove the feature with the lowest importance and so on, to realize the feature selection. The flowchart of LGBM's feature extraction is shown in Figure 2.

Here, we choose LGBM to reduce the input dimension of BP-NN. It not only can reduce the time for BP-NN training but also can reserve the features most correlated with the bioactivity value.

#### 3.2.2. BP-NN

*(1) BP-NN.* First, sum the weights of the input data *x*_1_, *x*_2_, *x*_3_, ⋯, *x*_*n*_ and then substitute the result value of the feedforward network as the independent variable value of this layer into the activation function of this layer *φ*(*v*)=ReLU(*v*); the output value can be expressed as follows:

(1) $$\begin{array}{c} \hat{y}=\text{ReLU}\left(\sum_{d=1,n=1}^{n}w_{d}x_{d}\right). \end{array}$$

Then, BP-NN needs to continuously adjust the weight parameter *w* based on feedforward and backpropagation to complete the learning process until the output is consistent with the actual value of the training sample. The weight adjustment formula is

(2) $$\begin{array}{c} w_{j}^{\left(k+1\right)}=w_{j}^{k}+\beta \left(y_{i}-\hat{y_{i}^{k}}\right)x_{ij}, \end{array}$$

where *w*^*k*^ is the weight of multiple inputs after passing through the *k*-th loop, *x*_*ij*_ is the *j*-th attribute's value of *x*_*i*_ in the training set, and the parameter *β* is the learning efficiency. If the actual value obtained is the same as the judgment value, then we can continue to call the existing method to predict the weight; if the actual value obtained is different from the judgment value, it means that there is a problem, and then a method needs to be redesigned to calculate weight and modify parameters.

The BP-NN method consists of some layers of the perceptron. The output of the perceptron is transformed by the ReLU function. The input dimension *k* of the first layer is determined by the number of molecular descriptors selected in Section 3.2.1. The input and output dimensions of the hidden layer are set to some value and the output dimension of the last layer is set to 1. The structure diagram of the BP-NN prediction method is shown in Figure 3.

*(2) BP-NN Evaluation Index.* The loss function of BP-NN uses *L*_1_loss, which refers to the average distance between the method predicted value $\hat{y}=\left(\hat{y_{1}},\hat{y_{2}},\ldots ,\hat{y_{n}}\right)$ and the true value *y*=(*y*_1_, *y*_2_,…, *y*_*n*_); it can be calculated as follows:

(3) $$\begin{array}{c} \text{loss}=\frac{\sum_{i=1}^{n}\left|\hat{y_{i}}-y_{i}\right|}{n}. \end{array}$$

We use the mean square error (MSE) to measure the BP-NN. The calculation of prediction accuracy also uses the *L*_1_ norm, which MSE can be calculated as follows:

(4) $$\begin{array}{c} \text{MSE}=\frac{1}{n}\sum_{i=1}^{n}{\left(\hat{y_{i}}-y_{i}\right)}^{2}, \end{array}$$

where *n* is the number of the test data, $\hat{y_{i}}$ is the predicted value, and *y*_*i*_ is the true value.

### 3.3. Prediction of ADMET Properties

#### 3.3.1. XGBoost

The extreme gradient boosting algorithm (XGBoost) is an integrated machine learning algorithm based on decision trees, using a gradient ascent framework, suitable for classification and regression problems, and used to solve supervised learning problems. Ensemble learning refers to the construction of multiple weak classifiers to predict the data set and then use a certain strategy to integrate the anticipated results of the multiple classifiers as the final prediction result [34]. It improves the traditional gradient boosting decision tree (GBDT) algorithm in terms of computing speed, generalization performance, and scalability.

Compared with gradient boosting, XGBoost introduces regularization in the loss function to establish the objective function:

(5) $$\begin{array}{c} J\left(\theta \right)=L\left(\theta \right)+\Omega \left(\theta \right), \end{array}$$

where

(6) $$\begin{array}{c} L\left(\theta \right)=\left({\hat{y}}_{j},y_{j}\right),\\ \Omega \left(\theta \right)=\gamma T+\frac{1}{2}\lambda {\|w\|}_{2}. \end{array}$$

As shown in (5), the objective function consists of two parts, *L*(*θ*) and Ω(*θ*), where *θ* represents various parameters learned from the given data. *L*(*θ*) is a differentiable convex loss function used to calculate the difference between the predicted result ${\hat{y}}_{j}$ and the target result *y*_*j*_. Generally, there are two commonly used loss functions, namely the mean square loss function $l\left({\hat{y}}_{j},y_{j}\right)=\left({\hat{y}}_{j},y_{j}\right){}^{2}$and the logistic loss function $l\left({\hat{y}}_{j},y_{j}\right)=y_{j}\ln\left(1+e^{-{\hat{y}}_{j}}\right)+\left(1-{\hat{y}}_{j}\right)\ln\ln\left(1+e^{{\hat{y}}_{j}}\right)$. This paper uses $l\left({\hat{y}}_{j},y_{j}\right)=\left({\hat{y}}_{j},y_{j}\right){}^{2}$ as the loss function [35]. Ω(*θ*) is a regularization term, which is used to punish the complexity of the method (i.e., the regression tree) [35]. Among them, *T* represents the number of leaves of the tree; *γ* represents the learning rate; and its value is between 0 and 1. *λ* is the regularization parameter; *w* is the leaf fraction; and *w*_*i*_ is the score of the ith leaf. Compared with the traditional GBDT algorithm, XGBoost uses 1/2*λ*‖*w*‖_2_, which can further avoid overfitting to strengthen the generalization ability of the method [36]. Given a data set with *n* samples and *M* characteristics, $D\;=\left\{\left(x_{\dot{j}},y_{j}\right)\right\}$, where $x_{\dot{j}}\left(j=1,2,\ldots ,n\right)$ represents a sample, *y*_*j*_ is the corresponding label, and *y* is the output of the method ${\hat{y}}_{j}$ is a set of *K* weak classifiers

(7) $$\begin{array}{c} {\hat{y}}_{j}=\varphi \left(x_{\dot{j}}\right)=\sum_{k=1}^{K}f_{k}\left(x_{\dot{j}}\right), \end{array}$$

where *f*_*k*_ represents the *k*-th weak classifier.

In addition, considering that (5) uses a function as a parameter and cannot optimize the space by the traditional method in Euclid, XGBoost accumulates the regression tree and appends a new optimization object in each iteration [37]. Therefore, at the *t*-th iteration, the objective function is defined as follows:

(8) $$\begin{array}{c} J^{\left(t\right)}=\sum_{j}^{N}l\left(y_{j},{\hat{y}}_{j}{}^{\left(t-1\right)}+f_{t}\left(x_{\dot{j}}\right)\right)+\Omega \left(f_{t}\right). \end{array}$$

In addition, XGBoost supports parallelization. It selects the best split point and performs parallel processing during enumeration, which greatly improves the efficiency of the algorithm and can be used in medicine prediction and screening.

#### 3.3.2. XGBoost Evaluation Index

This paper uses prediction accuracy and receiver operating characteristic (ROC) as evaluation indexes to evaluate XGBoost. ROC is present and expressed by the ROC curve.

For a binary classification problem, divide the instance into a positive class or a negative class; there will be four cases. If an instance is a positive class and is also predicted as a positive class, it is a true positive. If an instance is a negative class and is predicted as a positive class, it is called a false positive. Correspondingly, if the instance is a negative class and is predicted as a negative class, it is called a true negative, and if a positive class is predicted as a negative class, it is a false negative [38]. The contingency table of these four cases is shown in Table 2.

From the contingency table, the true positive rate (TPR) is introduced, and the calculation is

(9) $$\begin{array}{c} \text{TPR}=\frac{\text{TP}}{\left(\text{TP}+\text{FN}\right)}. \end{array}$$

Formula (9) refers to the proportion of positive examples identified by the classifier to all positive examples. The calculation for the false positive rate (FPR) is

(10) $$\begin{array}{c} \text{FPR}=\frac{\text{FP}}{\left(\text{FP}+\text{TN}\right)}. \end{array}$$

Formula (10) refers to the proportion of negative instances of the positive class that the classifier mistakenly believes to account for all negative instances. Then the calculation of prediction accuracy (PA) is

(11) $$\begin{array}{c} \text{PA}=\frac{\left(\text{TP}+\text{TN}\right)}{\left(\text{TP}+\text{FP}+\text{FN}+\text{TN}\right)}. \end{array}$$

The horizontal axis of the ROC curve is FPR, and the vertical axis is TPR. According to the actual situation, the ROC curve allows intermediate states, and the test results can be divided into multiple ordered categories, and then statistical analysis can be performed. Therefore, the ROC curve evaluation method is widely used in bioinformatics. We introduce area under roc curve (AUC) value to characterize the performance of the classifier. The AUC value is equal to the area enclosed by the ROC curve and the horizontal and vertical axis, usually between 0.5 and 1. The larger the AUC value, the better the comprehensive prediction performance.

### 3.4. BVAP-Pharmaceutical Product Candidates Screening

Based on the predicted bioactivity value and ADMET properties in Sections 3.2 and 3.3, we define the BVAP method to evaluate drug candidates. It is a weight calculation method. Users or experimenters can adjust the weight of bioactivity value and ADMET properties according to actual discovering needs. The calculation of BVAP is

(12) $$\begin{array}{c} \text{BVAP}=\alpha \text{BV}+\beta \text{AP,} \end{array}$$

where *α* is the weight of BV (i.e., bioactivity value) and *β* is the weight of AP (i.e., ADMET properties). As mentioned in Section 1, the ADMET properties include five kinds of properties, so we can detail the above calculation as follows:

(13) $$\begin{array}{c} \text{BVAP}=\alpha BV+\beta_{1}P_{1}+\beta_{2}P_{2}+\beta_{3}P_{3}+\beta_{4}P_{4}+\beta_{5}P_{5}, \end{array}$$

where *α* is the weight of BV and *β*_*i*_,  *i*=1,2,3,4,5 is the weight of the five kinds of AP. We can adjust the weights *α* and *β*_*i*_ to evaluate the drug candidates and then sort their BVAP values to get the best drug candidate.

## 4. Validation and Experiment

### 4.1. Data Set Preprocessing

The data set of compounds that antagonize the activity of Er*α* comes from question *D* of the 18th Chinese Graduate Mathematical Modeling Contest, which contains 729 molecular descriptors of 1,974 compounds, as well as the bioactivity value and ADMET properties of the compounds. The 1,974 compounds are the drug candidates that can antagonize breast cancer. The 729 molecular descriptors are a series of parameters used to describe the structural and property characteristics of Er*α*, including physicochemical properties (such as molecular weight, LogP, etc.), topological characteristics (such as the number of hydrogen bond donors, the number of hydrogen bond acceptors, etc.), and so on. The bioactivity value of Er*α* is usually expressed by pIC50, which is the experimental value. The larger the pIC50, the higher the bioactivity value. ADMET properties refer to good pharmacokinetic properties and safety in vivo. The related description of the data set is shown in Table 3.

In Table 3, there are four columns, and the first column is the compound molecular structure; the second column is the 729 molecular descriptors; and the third and the last columns are, respectively, the bioactivity value and ADMET properties. The molecular descriptors are equivalent to the features, and the bioactivity value and ADMET properties are the target value that needs to be predicted.

To facilitate modeling and prediction, this paper only considers the five ADMET properties of the compound in the data set, namely: (1) intestinal epithelial cell permeability (Caco-2), which can measure the ability of the compound to be absorbed by the human body; (2) cytochrome P450 enzyme (Cytochrome) P450, CYP3A4 subtype (CYP3A4), which is the main metabolic enzyme in the human body, which can measure the metabolic stability of compounds; (3) evaluation of compound cardiac safety (human ether-a-go-go-related gene, hERG), which can measure the cardiotoxicity of the compound; (4) human oral bioavailability (HOB), which can measure the proportion of the amount of medicine absorbed into the human blood circulation after entering the human body; and (5) micronucleus test (Micronucleus, MN), which is a method to detect whether the compound has genotoxicity [11, 38]. For the five ADMET properties, Caco-2: “1” represents the compound has better small intestinal epithelial cell permeability, and “0” represents the compound has poor small intestinal epithelial cell permeability; CYP3A4: “1” represents that CYP3A4 can metabolize the compound, and “0” represents that the compound cannot be metabolized by CYP3A4; hERG: “1” represents that the compound has cardiotoxicity, and “0” represents that the compound does not have cardiotoxicity; HOB: “1” means that the oral bioavailability of the compound is good, and “0” means that the oral bioavailability of the compound is poor; and MN: “1” means that the compound has genotoxicity, and “0” means that the compound is not genotoxic.

We first do data exploration and find that none of the molecular descriptors in the data set have null values, so there is no need to consider missing values. Then we preprocess 729 molecular descriptors. We set the variance *σ*=0.05 and the correlation coefficient *C*=0.95 through multiple experiments and validations. After data preprocessing (1) from Section 3.1, there are 361 remaining molecular descriptors. The correlation heat map is shown in Figure 4.

After data preprocessing (2) in Section 3.1, the number of molecular descriptors is reduced to 123.

### 4.2. Validation for Fusion Regression

In this part, we first split the data: 70% of them are used for training, 10% for validation to get the proper parameters, and 20% for testing. Also, the evaluation index MSE is got on the test data.

#### 4.2.1. LGBM for Feature Extraction

After Section 4.1, to make the BP-NN easy to train and more accurate, further feature extraction and dimensionality reduction can be performed to screen out the features related to the bioactivity value. LGBM is used to screen the top 20 molecular descriptors with higher importance degrees obtained on the training data, as shown in Figure 5.

It can be seen from Figure 5, according to the value of feature importance, we have screened out 20 molecular descriptors, which are “MDEC-23,” “LipoaffinityIndex,” “MLFER_A,” “maxHsOH,” “C1SP2,” “XLogP,” “BCUTp-1h,” “VC-3,” “TopoPSA,” “minHBa,” “WTPT-3,” “SCH- 7,” “MDEC-33,” “SHBint6,” “CrippenLogP,” “MDEC-22,” “BCUTp-1l,” “minHBint10,” “SHBint10,” and “MLogP.” Here, we choose the top 20 molecular descriptors because the competition data set tells us there are only 20 molecular descriptors that are most related to the bioactivity value.

#### 4.2.2. BP-NN

Based on the top 20 molecular descriptors in Section 4.2.1, we use the BP-NN to predict the bioactivity value.

By training and validation, we can decide and choose the best parameters for BP-NN. The BP-NN method consists of 1 input layer, 2 fully connected layers, and 1 output layer. The output of the perceptron is transformed by the ReLU function. The input dimension *k* of the first layer is set to 20 corresponding to the top 20 molecular descriptors. The input and output dimensions of the hidden layer are set to 300, and the output dimension of the last layer is set to 1. Among those hyperparameters, when the hyperparameter batch size is set to 2, 4, 8, and 16, the changes in the loss value are shown in Figure 6.

It can be seen from Figure 6 that when batch size is set to 2, the method can converge to a lower loss after 30 rounds of training. Through similar methods to filter other hyperparameters, a set of hyperparameters with relatively better final training effects is obtained, as shown in Table 4.

According to the obtained hyperparameters, the BP-NN is trained. Then the fusion regression assembles the LGBM for feature extraction and BP-NN, obtaining the MSE on the test data. The MSE is 1.1496, which can provide an effective method for the quantitative prediction of the bioactivity value.

### 4.3. Validation for XGBoost

In this part, we first split the data: 70% of them are used for training, 10% for validation to get the proper parameters, and 20% for tests. Also, the prediction accuracy and the ROC curve are both got on the test data.

#### 4.3.1. XGBoost

This paper uses XGBoost to predict the ADMET properties based on the preprocessed data in Section 4.1. The prediction accuracy of ADMET properties is shown in Table 5.

In Table 5, we get that the prediction accuracies of ADMET properties are 94.0% for Caco-2, 95.7% for CYP3A4, 89.4% for hERG, 88.6% for HOB, and 96.2% for MN.

### 4.4. Discussion

Alternatively, this paper uses another five methods mentioned in related work, which are SVM, RF, LDA, K-nearest neighbor (KNN), and naive Bayes (NB), to predict ADMET properties. The prediction accuracy of ADMET properties and the accuracy comparison with XGBoost is shown in Table 6.

The prediction accuracy of ADMET properties with the above five methods is compared with XGBoost used in this paper, as shown in Figure 7.

It can be seen from Figure 7 that the prediction accuracy of the XGBoost used in this paper for ADMET properties, which are Caco-2: 94.0%, CYP3A4: 95.7%, hERG: 89.4%, HOB: 88.6%, and MN: 96.2%, is higher compared with another five methods: SVM, RF, KNN, LDA, and NB. At the same time, we use the ROC curve to compare the comprehensive performance of the above six prediction methods. The comparison results are shown in Figure 8.

It can be seen from Figure 8, the AUC values of the XGBoost method used in this paper are: Caco-2: 0.933, CYP3A4: 0.954, hERG: 0.891, HOB: 0.839, and MN: 0.939, which are larger than the AUC values of another five methods. So the XGBoost has higher prediction accuracy and better performance.

### 4.5. Pharmaceutical Product Candidates Screening

According to the prediction results in Sections 4.2 and 4.3, we can use formula (12) to calculate the BVAP by setting proper weights. For example, if we set *α*=0.4, *β*_1_=0.1, *β*_2_=0.1, *β*_3_=0.1, *β*_4_=0.1, and *β*_5_=0.2, then we can get the screening list of the top 10 drug candidates in Table 7.

## 5. Conclusions

Aiming at the problem of drug discovery failure in the early stage of drug development due to low bioactivity value and poor ADMET properties, this paper proposes a screening model for pharmaceutical products candidates with better bioactivity value and ADMET properties and validates the data set of compounds that antagonize the activity of Er*α*. Firstly, data preprocessing is made in the data set for initial feature extraction; then the fusion regression is used to predict the bioactivity value, including LGBM for further feature extraction and the BP-NN method for bioactivity value prediction, and the MSE of fusion regression is 1.1496. Then the XGBoost is used to predict the ADMET properties, and the XGBoost prediction accuracy of ADMET properties are as follows: Caco-2: 94.0%, CYP3A4: 95.7%, hERG: 89.4%, HOB: 88.6%, and MN: 96.2%, and the AUC value are as follows: Caco-2: 0.933, CYP3A4: 0.954, hERG: 0.891, HOB: 0.839, and MN: 0.939. Finally, based on the predicted bioactivity value and ADMET properties, we use the BVAP method to screen the drug candidates with better bioactivity value and ADMET properties.

In summary, we make a difference in the prediction accuracy of ADMET properties compared with other methods, which is beneficial to improving the prediction and screening model for drug candidates. The prediction and screening model proposed in this paper has better comprehensive performance, which can also provide prediction services for the bioactivity value and ADMET properties.

While this paper also has some shortcomings: (1) the model proposed in this paper improves the problem of inaccurate prediction of ADMET properties but only extracts important features, but some properties are not considered. The next step will continue to expand the model. (2) The value or range of the molecular descriptor needs to be further verified after model expansion, and after that, a recommended reference value or range can be given.

Therefore, future work will be made to improve the above shortcomings.

## Figures and Tables

**Figure 1:** The pharmaceutical products screening model flowchart.

**Figure 2:** Flow chart of LGBM.

**Figure 3:** BP-NN method structure diagram.

**Figure 4:** Molecular descriptor correlation heat map.

**Figure 5:** LGBM feature extraction of the top 20 molecular descriptors.

**Figure 6:** The loss value of each training round.

**Figure 7:** Six methods' prediction accuracy of ADMET properties: XGBoost, SVM, RF, LDA, KNN, and NB.

**Figure 8:** Comparison of comprehensive performance of six prediction methods against five ADMET properties: (a) six prediction methods' ROC curve for Caco-2, (b) six prediction methods' ROC curve for CYP3A4, (c) six prediction methods' ROC curve for hERG, (d) six prediction methods' ROC curve for HOB, and (e) six prediction methods' ROC curve for MN.

**Table 1:** The advantages and disadvantages of SVM, RF, KNN, NB, LDA, and XGBoost.

Methods	Advantage	Disadvantage
SVM [16–19, 25, 29, 31]	SVM avoids the complexity of high-dimensional space and directly uses the kernel function of this space	SVM is difficult to implement for large training samples and determine the kernel function
RF [16, 19, 25–27, 31]	RF can handle very high-dimensional data without feature selection	RF may overfit on some noisy classification or regression problems
KNN [31]	The training time complexity of KNN is lower than the support vector machine (SVM)	The amount of calculation is large
	Compared with naive Bayes (NB), it has no assumptions about the data, has high accuracy, and is insensitive to outliers	When the sample is unbalanced, the prediction accuracy of rare categories is low
NB [16, 32]	NB performs well on small-scale data, and the algorithm is relatively simple	The posterior probability is determined by the prior and the data, and then to determine the classification, so there is a certain error rate in the classification decision
LDA [16, 26]	LDA works better when the sample classification information depends on the mean rather than the variance	LDA is not suitable for dimensionality reduction of samples from non-Gaussian distributions and may overfit
XGBoost [31]	Regularization is added to the loss function to prevent overfitting	The split gain of many leaf nodes at the same level is low, and it is unnecessary to perform further splits, which may bring unnecessary overhead
	Parallel computing makes the algorithm more efficient	
	Memory optimization	

**Table 2:** The contingency table of the four cases.

	Predict			
		1	0	Sum
True value	1	TP	FN	Actual positive (TP + FN)
	0	FP	TN	Actual negative (FP + TN)
Sum		TP + FP	FN + TN	TP + FP + FN + TN

**Table 3:** Data set description.

SMILES	nAcid ALogP … AMR	pIC50	ADMET
Compounds' structure	Molecular descriptors	Bioactivity value	Absorption, distribution, metabolism, excretion, toxicity

**Table 4:** BP-NN method's hyperparameter values.

Hyperparameter	Value
Learning rate (LR)	0.001
Batch size (batch_size)	2
Number of training rounds (epochs)	30

**Table 5:** The prediction accuracy of ADMET properties.

ADMET properties	Prediction accuracy (%)
Caco-2	94.0
CYP3A4	95.7
hERG	89.4
HOB	88.6
MN	96.2

**Table 6:** The prediction accuracy of another five prediction methods and the accuracy comparison with XGBoost.

Prediction methods	ADMET properties	Prediction accuracy (%)	Accuracy improvement (%)
SVM	Caco-2	86.8	7.2
	CYP3A4	87.6	7.8
	hERG	86.3	3.1
	HOB	87.3	1.6
	MN	85.8	10.4

RF	Caco-2	93.2	0.8
	CYP3A4	94.2	1.5
	hERG	88.1	1.3
	HOB	88.4	0.5
	MN	94.9	1.3

LDA	Caco-2	88.5	5.5
	CYP3A4	93.2	2.5
	hERG	86.1	3.3
	HOB	85.3	3.6
	MN	87.6	8.6

KNN	Caco-2	85.6	8.4
	CYP3A4	87.9	7.8
	hERG	80.5	8.9
	HOB	74.2	14.7
	MN	81.0	15.2

NB	Caco2	82.5	11.5
	CYP34	85.6	10.1
	hERG	744	15
	HOB	56.5	32.4
	MN	72.4	23.8

**Table 7:** The screening list of top 10 drug candidates.

SMILES (drug candidates)	BV	*P*1	*P*2	*P*3	*P*4	*P*5	BVAP
C[C@@H]1Cc2c([nH]c3ccccc23)[C@H](N1CC(C) (C)F)c4c(F)cc(\C=C\C(=O)O)cc4F	9.860	1	1	1	1	1	4.544048
Oc1ccc2c(C(=O)c3ccc(OCCN4CCCCC4)cc3)c(sc2c1)c5ccc(Cl)cc5	10.337	0	1	1	0	1	4.534897
COc1ccc(C2=C(c3ccc(O[C@H]4CCN(CCCF)C4)cc3)c5ccc(O)cc5CCC2)c(C)c1	9.699	1	1	1	0	1	4.379588
Oc1ccc(cc1)c2sc3cc(O)ccc3c2C(=O)c4ccc(cc4)N5CCN(CC5)c6ccc(Cl)cc6	9.658	0	1	1	1	1	4.363031
CC(C)N1CCN(CC1)c2ccc(cc2)C(=O)c3c(sc4cc(O)ccc34)c5ccc(O)cc5	9.553	0	1	1	1	1	4.321137
OC1CCC(CC1)C2=C(c3ccc(O[C@H]4CCN(CCCF)C4)cc3)c5ccc(O)cc5CCC2	9.699	0	1	1	0	1	4.279588
Oc1ccc2C(=C(CCCc2c1F)c3ccc(OC(F)F)cc3F)c4ccc(O[C@H]5CCN(CCCF)C5)cc4	9.699	0	1	1	0	1	4.279588
C[C@@H](COc1ccc(cc1)C2Oc3ccc(O)cc3C(=C2c4cccc(O)c4)C)N5CCCCC5	9.699	0	1	1	0	1	4.279588
C[C@@H](COc1ccc(cc1)C2Oc3ccc(O)cc3C(=C2c4cccc(O)c4)C)N5CCCCCC5	9.699	0	1	1	0	1	4.279588
C[C@H](CF)CN1[C@H](C)Cc2cc(O)ccc2[C@H]1c3c(F)cc(\C=C\C(=O)O)cc3F	9.432	1	1	1	0	1	4.272719

## Data Availability

The dataset sources are from D Question of the 18th China Postgraduate Mathematical Contest in Modeling.
